The article "Development of NLP-Integrated Intelligent Web System for E-Mental Health" was retracted in 2023. Reasons: signs of a paper mill; compromised peer review; unreliable results or conclusions.

# Development of NLP-Integrated Intelligent Web System for E-Mental Health

**DOI:** 10.1155/2021/1546343

**Published:** 2021-12-13

**Authors:** Abid Hassan, M. D. Iftekhar Ali, Rifat Ahammed, Sami Bourouis, Mohammad Monirujjaman Khan

**Affiliations:** ^1^Department of Electrical and Computer Engineering, North South University, Bashundhara, Dhaka, 1229, Bangladesh; ^2^Department of Information Technology, College of Computers and Information Technology, Taif University, P.O. Box 11099, Taif 21944, Saudi Arabia

## Abstract

As the COVID-19 pandemic continues, the need for a better health care facility is highlighted more than ever. Besides physical health, mental health conditions have become a significant concern. Unfortunately, there are few opportunities for people to receive mental health care. There are inadequate facilities for seeking mental health support even in big cities, let alone remote areas. This paper presents the structure and implementation procedures for a mental health support system combining technology and professionals. The system is a web platform where mental health seekers can register and use functionalities like NLP-based chatbot for personality assessment, chatting with like-minded people, and one-to-one video conferencing with a mental health professional. The video calling feature of the system has emotion detection capabilities using computer vision. The system also includes downloadable prescription facilities and a payment gateway for secure transactions. From a technological aspect, the conversational NLP-based chatbot and computer vision-powered video calling are the system's most important features. The system has a documentation facility to analyze the mental health condition over time. The web platform is built using React.js for the frontend and Express.js for the backend. MongoDB is used as the database of the platform. The NLP chatbot is built on a three-layered deep neural network model that is programmed in the Python language and uses the NLTK, TensorFlow, and Keras sequential API. Video conference is one of the most important features of the platform. To create the video calling feature, Express.js, Socket.io, and Socket.io-client have been used. The emotion detection feature is implemented on video conferences using computer vision, Haar Cascade, and TensorFlow. All the implemented features are tested and work fine. The targeted users for the platform are teenagers, youth, and the middle-aged population. Mental health-seeking is still considered taboo in some societies today. Apart from basic established facilities, this social dilemma of undergoing treatment for mental health is causing severe damage to individuals. A solution to this problem can be a remote platform for mental health support. With this goal in mind, this system is designed to provide mental health support to people remotely from anywhere worldwide.

The article "Development of NLP-Integrated Intelligent Web System for E-Mental Health" was retracted in 2023. Reasons: signs of a paper mill; compromised peer review; unreliable results or conclusions.

## 1. Introduction

The whole world is going through the COVID-19 pandemic. Approximately 3.46 million people have died, and many are waiting in line. Almost every country in the world has gone through some lockdown. This whole situation has severely affected people's mental health. COVID-19 home confinement had a detrimental effect on mental wellbeing and emotional status, with more people reporting low mental wellbeing (+12.89%), (ii) feeling dissatisfied (+16.5%), (iii) developing depression (+10%), and (iv) a need for psychosocial help (+16.1%) than “before” the confinement period [1]. According to the World Health Organization, mental health is a condition of wellbeing in which an individual accepts his or her abilities, can cope with everyday stressors, can work productively and fruitfully, and can contribute to his or her community. Mental health encompasses physical, financial, and social wellbeing. It has an impact on people's thoughts, feelings, and behaviors. It also has an effect on how people manage stress, socialize, and make choices. Every stage of life, including childhood, adolescence, and maturity, requires mental wellness. Though mental health is an essential aspect of life, it is often overlooked. Globally, almost 970 million people are suffering from mental health issues. In Bangladesh, over 7 million individuals suffer from anxiety and depression disorders [2]. An estimated 10,167 people died by suicide in 2012, with 4% of males and 6% of females aged 13-17 years contemplating suicide [2]. Depression, stress, and anxiety levels in Bangladesh have been found to be as high as 54.3%, 59.0%, and 64.8%, respectively [3].

Out of many reasons, one of the most prominent obstacles for addressing mental health conditions is the availability of professional help. As a 3rd world country, Bangladesh has poor health infrastructure where essential medical assistance is not always accessible. In such circumstances, seeking professional help for mental health conditions is quickly overshadowed. Again, the social structure is often not that open-minded even today to accept visiting doctors or professionals for mental health support. The situation is even worse in village areas. And sometimes the external conditions create obstacles. People are less likely to visit a mental health professional in a crowded country like Bangladesh, where traffic jams are a serious issue. Telemental health facilities can be the best solution considering all the obstacles present for seeking mental health. As mental health treatment rarely needs any heavy machinery, telemental health support can be a very useful solution.

The article "Development of NLP-Integrated Intelligent Web System for E-Mental Health" was retracted in 2023. Reasons: signs of a paper mill; compromised peer review; unreliable results or conclusions.

Some existing systems for mental health and support are already out there. The first one is the “MonerBondhu Wellbeing Center” [4]. They provide support for distress via a helpline number and provide a free course to better health. The second one is “Therapy Route” [5]. They are a search engine to search mental therapists within any area or city. Then, the other one is “Let's Talk BD” [6], which offers virtual counseling sessions online. The existing systems for mental health care provide some shared facilities. They are arranging counseling sessions with psychiatrists. Besides, some of them have volunteers to hear users' conversations. The web platform presented in this paper is also a telemental health platform. However, the platform presented uses more technically advanced assessment tools to obtain data for mental health analysis. This system uses NLP-based conversational chatbots for health seekers to primarily assess themselves with personality tests. The video conference, which is the main part of any conventional telehealth system, is also present in the system but with more power, as it has emotion detection functionality using computer vision. There is a large body of research that supports the use of NLP and computer vision for mental analysis.

Natural language processing (NLP) is an essential branch of artificial intelligence (AI) that studies the interactions between humans and computers via natural language [7]. Natural language processing or NLP combines computer science, artificial intelligence, and linguistics, which deals with human language and computer interaction. NLP is the system of processing and analyzing large amounts of natural language data. NLP is not a new concept. NPL's history can be divided into three stages: symbolic NLP, statistical NLP, and neural NLP are the three types of NLP.

Neural NLP is the present form of NLP used for natural language processing with representation and machine learning capabilities. NLP was enriched at a large scale with AI capabilities after 2010. In [8], the authors showed that, following the success of deep learning in object recognition with ImageNet, deep learning approaches were added to NLP in 2012. In [9], the authors present that significant technological improvements have also come in speech recognition with switchboards. Deep learning techniques outperformed statistical learning methods with surprisingly better results in a short period. As of now, the neural network-based NLP framework (referred to as “neural NLP” hereafter) has reached new levels of quality and has established itself as the dominant approach for NLP tasks such as machine translation (MT), machine reading comprehension (MRC), and chatbots. People's texts are automatically processed when they write digitally (e.g., email or social media). Natural language processing (NLP) techniques infer what people say and feel, and these inferences can be used to send messages or take other actions. In [10], the authors state that one of the most common applications of NLP is in marketing, where companies use it to analyze emails and social media to create targeted ads that can influence people to make decisions on buying something. On the other hand, NLP methods have applications that go beyond marketing. For example, NLP methods have been recognized as a key area of development within artificial intelligence (AI) in the medical community [11]. There has been significant use of conversational NLP in the construction of chatbots. Some researchers have classified them into two categories: social chatbots and task-oriented chatbots [12]. Social chatbots were made to carry out conversions like humans. The term chit-chat is sometimes used for addressing them. Task-oriented chatbots can be classified as either general task-oriented or special task-oriented. The system uses a special task-oriented chatbot to figure out the mental distress of the help seekers. There are some popular approaches to creating a chatbot. These include rule-based chatbots, sequence-to-sequence learning, data-driven chatbots, information retrieval chatbots, machine learning-based chatbots, and reinforcement learning.

The article "Development of NLP-Integrated Intelligent Web System for E-Mental Health" was retracted in 2023. Reasons: signs of a paper mill; compromised peer review; unreliable results or conclusions.

Apart from these approaches, hybrid methods are also popular, which are a combination of these approaches. The Alibaba shopping chatbot is a hybrid chat that follows a hybrid approach to information retrieval and a sequence-to-sequence learning approach [13]. Chatbot evaluation is one of the most important aspects of it. Out of many ways, evaluation by humans is the method with the highest quality. Nevertheless, it is very costly. In [14], the authors show that some IR-based chatbots can be evaluated using basic accuracy and recall metrics to function as search engines. Automatic evaluation techniques, such as BLEU, have recently been tested. In [15], the authors presented ROUGE, which is also another example. These are used for text summarization and automatic transitions of texts. These metrics calculate the *n*-gram overlap between a system's output and a set of references. These metrics were used to compare chatbot responses to human responses to the same question when evaluating chatbots. In evaluating dialogue systems, *N*-gram overlap-based metrics have limitations because two answers can be completely different but have the same meaning. Chatbots have also been evaluated using perplexity [16]. Perplexity is a metric that measures how well a language model predicts the likelihood of words in a test set. It was first used to assess language models. So, for a conversational NLP-based chatbot, a hybrid approach and solid evaluation methods need to be implanted to ensure it is not just a redundant feature.

The article "Development of NLP-Integrated Intelligent Web System for E-Mental Health" was retracted in 2023. Reasons: signs of a paper mill; compromised peer review; unreliable results or conclusions.

Computer vision is a branch of artificial intelligence that teaches computers to read, understand, and interpret images. Machines can use digital photos, videos, and deep learning models to detect and classify objects and then respond to what they see. It is a multidisciplinary research framework for analyzing how machines can comprehend digital pictures or videos at a high level. From an engineering perspective, it is aimed at comprehending and automating tasks that the human visual system is capable of doing. The usage of computer vision for emotion detection from facial expressions is quite a new field of interest for researchers. In [17], researchers state that one of the most important aspects of human emotion recognition is facial expression. According to Li and Jain, it can be defined as expressive shifts in response to a person's inner mental state, ideas, or social interactions [18]. Much work has recently been done in the fields of facial expression recognition studies [19, 20]. Convolutional neural networks- (CNN-) based face recognition algorithms are quite popular currently [21]. As computer vision is a broad field, researchers have taken different approaches to introducing a computer vision-based system of this kind. In [22], a researcher from Indiana University have used autoencoders in the first method to create a unique representation of each emotion, while an 8-layer convolutional neural network is used in the second method (CNN). The JAFFE posed-emotion dataset was used to train these approaches, and their robustness was tested on 100 random photos from the Labeled Faces in the Wild (LFW) dataset, which contains candid rather than posed photos. The findings indicate that with additional fine-tuning and depth, the CNN model can outperform state-of-the-art approaches for emotion recognition.

Researchers from the Federal University of Esparto Santo published a convolutional network-based facial recognition system in [23]. In this research, they suggest a straightforward approach for face emotion identification that combines traditional techniques like convolutional networks with image preprocessing procedures. Depending on the feature set, convolutional networks and most machine learning methods achieve better accuracy. They have distributed their work in a few steps that go as (1) spatial normalization, (2) synthetic sample generation, (3) image cropping, (4) downsampling, (5) intensity normalization, and (6) convolutional network. In [24], researchers studied mental health using data from numerous trusted sources such as MEDLINE, medRxiv, Web of Science, PubMed, Web of Science Who database, and Oxford COVID-19 tracker database. They, in total, assessed 226,638 individuals through 60 studies. During the COVID-19 pandemic, the global prevalence of depression and anxiety was 24% and 21%, respectively.

The article "Development of NLP-Integrated Intelligent Web System for E-Mental Health" was retracted in 2023. Reasons: signs of a paper mill; compromised peer review; unreliable results or conclusions.

The studies presented above demonstrate that conversational NLP and computer vision can be used for mental health analysis, but they do not focus on a platform that can help people in mental distress. These systems are very good at displaying the capabilities of NLP and computer vision technologies but lack a user-friendly model. Considering the capabilities of NLP and computer vision, a user-friendly platform for mental health detection and support is presented in this paper.

The “MonerBondhu Wellbeing Center” [4] does not offer video calling. It only provides facilities for teletherapy through voice calls and provides a free online course. The system presented in this paper is more advanced, with a video calling feature with professionals. “Therapy Route” [5] is basically a search engine for finding psychiatrists. The system in this paper is well equipped with this finding psychiatrist feature. “Let's Talk BD” [6] is another mental health-seeking platform that is available in Bangladesh. Though it has teletherapy and video calling features, it does not provide emotion detection on video calls or conversational NLP chatbots, which are present in the system presented in this paper. The dataset used in the implementation is novel which is constructed using the Myers-Briggs Type Indicator or MBTI personality test cases. So, it can be said that the system presented in this paper is way more advanced and novel than the state-of-the-art systems that are available in the niche of telemental health.

The objective of this study is to develop an NLP-integrated intelligent web system for e-mental health. This paper presents a web-based mental health support system. On this platform, people will seek mental health support remotely without needing to step outside of their houses. At first, users will be authenticated with the necessary information. Then, they will be able to use this interactive conversational NLP-based chatbot. This chatbot will be the primary assessment tool to determine mental health conditions through psychological experiments that experts have designed. These assessments will filter the users into groups where the group members will have the option to sit in a conference through the system to share their feelings. These group talks are very relieving for highly depressed and suicidal people. A mental health support expert will join their conference and assess the mental help seekers. Then, for the final assessment, the help seekers will sit for one-to-one meetings with a mental health expert. In this stage, computer vision compatibility of the system will help the expert analyze help seekers' condition from the individual facial expression. The experts will be facilitated with proper documentation methods, and the results will be shown as progress reports.

The article "Development of NLP-Integrated Intelligent Web System for E-Mental Health" was retracted in 2023. Reasons: signs of a paper mill; compromised peer review; unreliable results or conclusions.

The main motivation of the study is to provide a remote, one-stop solution for everyone to take care of their mental health as it is one of the most deprived sectors in healthcare. In our country, people feel shy about their mental health, which seems taboo in our society. So, people often do not want to go to any mental health care center to take any counseling session from any mental health expert, and they keep raising their problems further. Using this mental health care platform, anyone can take care of his mental health without any hassle and hesitation because he can get all the facilities here. Going out for a counseling session and waiting for an appointment with any psychiatrist is a very time-consuming fact. Any user can get help without going out and a long wait for an appointment on this platform. Moreover, this service provides everything in one place, so the user can also save his money without going to different mental health clinics to get the services.

In Section 1, the introduction has been discussed.  Section 2 provides the methods and materials. System modules are introduced in Section 3.  Section 4 describes the results and analysis. Finally, a conclusion is provided in Section 5.

## 2. Methods and Materials

The methods and resources used in this system for building a mental health care system using conversational NLP and computer vision are discussed in this part. The system consists of three subsystems, conversational NLP chatbot, video conference, and web forum. All three subsystems have their purpose with distinct methodologies and results. The combined result of all three subsystems is stored as “user data” in the system's central database. The first subsection displays an overall system diagram. After that, the subsections present the chatbot, video calling, and web forum subsystem, respectively. Finally, it concludes with a use case diagram of the whole system.

The article "Development of NLP-Integrated Intelligent Web System for E-Mental Health" was retracted in 2023. Reasons: signs of a paper mill; compromised peer review; unreliable results or conclusions.

In the first part of this chapter, the whole system diagram is shown and described. Then, all the subsystems are focused on with their corresponding diagrams. Lastly, the use case diagram is described as well.

### 2.1. The System Diagram

Figure 1 indicates the whole system flowchart with three vital subsystems. The stakeholders will be categorized into three types by authentication. They will be the regular users or the patients, the psychologists, and the admins. After going through authentication, they will have access to the “web forum,” which is the center of the whole system. Besides, there is a subsystem that only patient users will face, which is the “conversational AI chatbot,” which will evaluate their states and categorize them in their category. This chatbot subsystem is one of the vital subsystems. Meanwhile, in the web forum, regular events will happen as it happens in a forum. People will be able to use different features, such as creating posts, commenting on them, and asking for help.

Apart from all the activities happening in the web forum, there will be regularly scheduled video conference calls between the users and the psychologists. They will sit face-to-face on the video call, talk about issues, and do tests as they wish. This subsystem is going to have the emotion recognition feature. When the user is talking to the psychologists, the module will try to track and recognize the user's facial expression and capture the emotion, which will certainly help further analysis and tests upon them. All the relevant information and statistics will be stored in the central database.

### 2.2. The Chatbot Subsystem

Figure 2 shows the focused view of the chatbot subsystem. This subsystem is one of the vital features of the whole system. The specialty is that it is built as a “data retrieval conversational chatbot” based on natural language processing. This subsystem has a novel dataset with over 150 conversation phrases which makes it efficient to evaluate one's mental state correctly. After evaluating the user's state, it will categorize him, which will cause the user to find his relevant posts or information that might help him regarding his mental state.

### 2.3. The Video Call Subsystem

Figure 3 focuses on the significant video call subsystem diagram. In this subsystem, the user can connect to a psychologist using their IDs. This feature will be integrated into the main website, as users will have regularly scheduled meetings with the psychologists. There they will talk about their issues and get assessed by different tests conducted by the psychologists. The vital feature of the subsystem is the emotion recognition feature. When conducting the session, the user's facial expression will be monitored. This module is a computer vision model trained with datasets featuring people's expressions and emotions. Both the manual data from the psychologists and the automated data from that computer vision model will be stored in the central database for further analysis and tests.

The article "Development of NLP-Integrated Intelligent Web System for E-Mental Health" was retracted in 2023. Reasons: signs of a paper mill; compromised peer review; unreliable results or conclusions.

### 2.4. The Web Forum Subsystem

Figure 4 shows the basic web forum subsystem, which is the heart of the whole system. Here, all the human interaction happens. This can be said as a portal to all the subsystems as well. All the users, along with the psychologists and admin, will be able to post relevant “blog threads” related to mental health and issues. They can comment or reply on those threads if they want. The psychologists and the admins have access to the patient's profile to see their state at that moment and the progress they are making with all the necessary records. This module is significant as it holds and controls the whole structure along with the subsystem to make the whole scenario efficient.

### 2.5. Use Case Diagram

Figure 5 focuses on the use case diagram for the system. The stakeholders of this system are regular users/patients, psychologists, and admins/moderators. All the users, including patients, psychologists, and admins, will go through the authentication process to get access to the web forum and all other subsystems. Only patient users will be assessed through the chatbot. Again, all users will be able to create blog posts and comment on the web forum. The direct face-to-face interaction between the patient and the psychologist happens in the video conference use case. All of them can see users' profiles, but only the psychologists and admin can see the records. Only the admins are going to have access to see the psychologists' profiles and do CRUD operations over the users' and psychologists' lists.

## 3. System Modules

The system has three main modules. They are the NLP chatbot, the video conference, and the emotion detection module. Different technologies have been used to make the modules as per the system's needs.

### 3.1. NLP Conversational Chatbot

A chatbot is a system with artificial intelligence that can interact with people [23]. This chatbot module of this paper works as the primary assessment tool for mental health analysis. In this chatbot, MBTI test cases have been used to assess a person's mentality. The four bipolar psychological dimensions measured by the MBTI (P) are introvert (I) versus extravert (E), sensing (S) versus intuition (N), thinking (T) versus feeling (F), and judging (J) versus perceiving (P) [24]. The MBTI assigns each person a four-letter type that reflects their preferences in each category. The chatbot can assess a person's mentality through various psychological preferences in how people perceive the environment and make decisions through dialogue. This deep neural network-based chatbot works as the primary filtering tool and can be divided into groups to provide them with proper mental support.

The article "Development of NLP-Integrated Intelligent Web System for E-Mental Health" was retracted in 2023. Reasons: signs of a paper mill; compromised peer review; unreliable results or conclusions.

#### 3.1.1. Technologies Used

- Python
- Keras
- TensorFlow
- Natural Language Toolkit (NLTK)
- Long Short-Term Memory (LSTM)

#### 3.1.2. Description of Technologies

The language used for coding the chatbot is Python. Several python packages have been imported as per the module's requirement. The algorithm used for the deep neural network chatbot is LSTM. LSTM networks are a sort of recurrent neural network that can learn order dependence in sequence prediction challenges. The Natural Language Toolkit (NLTK) is a Python programming platform for statistical natural language processing that interacts with human language input (NLP). It includes text processing tools for tokenization, parsing, categorization, stemming, tagging, and semantic reasoning. A JSON formatted MBTI dataset has been used in this paper. JSON is an open standard file format and data exchange format that uses human-readable text to store and transfer data objects such as attribute-value pairs and arrays (or other serializable values). It is a basic data format that can accommodate a wide range of data transfers, including communication between web apps and servers. The data saved in the JSON dataset has been deserialized using the Pickle Module of Python. Pickle is a Python library for serializing and deserializing Python object structures. To put it differently, it is the process of converting a Python object into a byte stream in order to save it to a file/database, preserve program state between sessions, or send data over the network.

The Keras API is used in this paper to provide a Python interface for the module. It acts as an interface to the TensorFlow library. The Keras sequential model has been used here. Also, dense, activation, and dropout layers are imported into the paper. In this module, Keras' SGD class created a stochastic gradient descent optimizer with a learning rate and momentum.

#### 3.1.3. Implementation

The chatbot works as the primary assessment tool in this paper. A registered user can chat with a chatbot from our web app. Through conversational assessment, the chat asks different questions based on MBTI test cases.

The main file for the module creates essential packages (NLTK, JSON, Pickle, and Keras) for importation. The dataset is tokenized for each word and lemmatized to remove every duplicate word from the list. Lemmatizing is the process of translating a word into its lemma form and then saving the Python objects. It will be used during prediction in a pickle file and to create a numbered training dataset that is understood by the computers.

The article "Development of NLP-Integrated Intelligent Web System for E-Mental Health" was retracted in 2023. Reasons: signs of a paper mill; compromised peer review; unreliable results or conclusions.

As soon as the training data is ready, the deep neural network with three layers, dense, activation, and dropout, is created using the Keras sequential API. The training is conducted for 30 epochs. As the training completes the epoch cycles, the Graphical User Interface (GUI) chatbot module is able to have a conversation and respond accordingly.

### 3.2. Real-Time Communication Module

In the web application system, there are going to be two real-time communication systems fully dedicated to the users. This will make it easier for the patient to get help with their psychological state by communicating with peers and, in a special case, to get help from a psychiatrist. These systems are fully integrated within the web app so that it will act as a complete hub and be user-friendly for everyone to get all kinds of help and everything under a single platform.

The real-time modules are

1. real-time chatting forum (user to user, user to psychiatrists, and psychiatrists to psychiatrists)
2. user to psychiatrists: a real-time video call system (user to psychiatrists)

#### 3.2.1. The Module's Purpose

The entire paper is centered on the patient's wellbeing and treatment for psychological issues. Communication is an important aspect of psychiatric care and one of the fundamental competencies. It allows for safe and high-quality patient treatment [25]. It has also been found that health care errors are often connected with poor communication. During the COVID-19 lockdown situation, this has gone worse. The gap has been increased, especially between the patients dealing with psychological issues and the psychiatrists. To decrease the gap and deal with distance maintenance, this module has been decided to be introduced under a single shed along with other relevant features.

The chat forum has the aim of letting all the users talk, share information, help each other out when they need help, etc. The users will also be able to talk to any psychiatrist by text chat in a designated chat channel. There are going to be multiple chat channels for multiple purposes. One will be able to join a specific chat channel depending on his or her needs.

Another real-time module is the video call system. This is also an integrated real-time communication service of the web app. It has a specific and restricted aim, which is to enable a user and psychiatrist to communicate during their scheduled meeting time. A psychiatrist will give the scheduled patient a code to join in a video call. Talking face-to-face is very vital for dealing with psychological issues. Online therapy is not as good as talking face-to-face with a psychiatrist or a clinician. So, this module has been introduced along with others, under a single hood to make it easier for both parties. The video conference is also not as efficient as physically attending a face-to-face session, but this recent situation has made it an essential service.

The article "Development of NLP-Integrated Intelligent Web System for E-Mental Health" was retracted in 2023. Reasons: signs of a paper mill; compromised peer review; unreliable results or conclusions.

#### 3.2.2. Technologies Used in the Module

To get the whole technical part of this module done, socket programming has been used. Socket programming is basically the way to connect two or multiple nodes on a network to communicate with each other. To make this happen, the following modules have been used.

1. Express.js
2. Socket.io
3. Socket.io-client

Express.js is a backend framework for Node.js, which has been used to build the backend of our system. In this backend system, the real-time modules have been built. To implement both the real-time chat and video system, Socket.io has been used. Socket.io is a popular open-source library, which serves the purpose of real-time web applications. It enables real-time, bidirectional communication between web clients and servers. This library is based on the WebSockets API, which actually allows you to make connections between server and client. On the other hand, the Socket.io-client is responsible for receiving emitted data on the client side from the server side and making it client side-friendly.

#### 3.2.3. Implementation of the Technologies in the Module

*(1) Frontend*. To make the frontend section of this real-time communication part of the web app, React.js along with Socket.io-client has been used. This part with the main frontend part runs separately from the backend system. This part basically receives the emitted data and also sends input from the client side to the server.

In Figure 6, it can be seen that every time the video call page loads in the web app, it will try to get video and audio access from the client device. The stream window screen will be detected as a stream object to be delivered to the server side. Along with this, it will objectify the user as well, allowing him to receive and make a call.

Figures 7 and 8 show the functions for making and receiving calls in the system, respectively.

The client side for the chat module follows the same structure.

*(2) Backend*. The backend system is a web server based on Node.js built with the help of the Express.js framework. The whole system backend is integrated here along with the real-time module backend. With the help of the Socket.io library, the communication server is built.

The article "Development of NLP-Integrated Intelligent Web System for E-Mental Health" was retracted in 2023. Reasons: signs of a paper mill; compromised peer review; unreliable results or conclusions.

Figure 9 shows the method of a user getting connected to a chat room on a successful connection.

Figure 10 shows the way the backend listens to chat messages which are later delivered to the frontend for it to receive and render on the client side.

Figure 11 shows the backend configuration and the impacts of the actions taken on the client side regarding calling, answering, and disconnecting a call.

### 3.3. Emotion Detection Module Using Computer Vision

We aim to detect patients' emotions by using this facial emotion detection technology. It will help the doctors to prescribe medicines more precisely. If the doctor can visually identify the emotional disturbance of the patient, he can give better treatment. Moreover, it will become easier for a consultant to reevaluate the problems of the patient as the system can detect the facial expressions more accurately. We believe this technology can bring a remarkable change in the mental illness sector.

#### 3.3.1. Technology Used

- Computer vision
- Haar Cascade
- Keras
- TensorFlow

#### 3.3.2. Technology Brief

OpenCV is the open-source Computer Vision Library, which is developed by Intel. Keras is an open-source Python library which is actually used for developing and evaluating deep learning models. TensorFlow is an end-to-end free open-source symbolic math library based on data flow for machine learning and artificial intelligence. Haar Cascade is an algorithm of object detection, which can identify faces in an image or a video running in real time, which can be accessed with OpenCV methods.

#### 3.3.3. Technology Implementation

During the video conference with the doctor for the emotion detection part, we use computer vision to execute this artificial intelligence part.

In this whole process, we actually followed 3 steps to execute the detection part. These are

- collecting datasets for various emotions
- deep learning for training the model
- using the model to predict the proper emotion

First, for creating the dataset, we created a total of five classes for five vital emotions. They are neutral, happy, sad, angry, and surprise.

In the training part, we use three simple steps.

- Import some required libraries
- Use images and labels to train the model
- Train the model by using Keras and TensorFlow on those given parameters

And in the final detection part, we go through these steps.

Firstly, we will collect the live video or the recorded video of the user end, which is actually some continuous frames of the user face.

After that, we use the XML file named “haarcascade_frontalface_default,” which is a face classifier, to detect the user's face.

The article "Development of NLP-Integrated Intelligent Web System for E-Mental Health" was retracted in 2023. Reasons: signs of a paper mill; compromised peer review; unreliable results or conclusions.

Then, we will go through the h5 file named “Emotion_Detection” to detect and declare the emotion label, which is actually the storage of the Keras trained model.

## 4. Results and Analysis

In this chapter, the major features of the website will be analyzed, along with the basic website systems. The results of the system features will be analyzed as results and will be compared to existing systems.

### 4.1. Home Interface

Figure 12 shows the home interface of the web forum subsystem's home interface. It can be called the portal to the other features in the paper. Users will be able to post, comment, contribute, and so on. It will also navigate them to the other features. In the landing and subpage interfaces, users can go through many online tests and surveys from different sites and have all those options in one place. Very important information is provided and video tutorials, such as yoga, breathing exercises, and some relaxation music. The frontend technologies used here are HTML, Cascading Style Sheets (CSS), and the React.js library. React.js is a JavaScript library for building reusable User Interface (UI) components. React.js is used here for its component reusability, so it does not have to render duplicate HTML codes and keep everything efficient. Using React.js on the website, data can be changed without even reloading the website. The main purpose of using this technology is to make it fast, scalable, and simple.

### 4.2. Login and Authentication

Authentication is a vital part of every website system. In this system, there are two categories of authentication systems. One is for the regular user or patient, and the other one is for psychologists. Both of the authentication systems are controlled by Google Firebase. There is a regular login feature with email and password, and an OAuth feature has also been implemented for a more user-friendly and secure authentication process.

Figure 13 shows the login/authentication system for psychologists. They have to provide additional NID and their professional registration number to get authenticated as a psychologist. If they use the OAuth process, they have to provide the additional NID and registration number later for the special access as a psychologist.  Figure 14 shows the regular authentication process for the patients.

### 4.3. Prescription Page

The registered psychiatrist will have their own authenticated private route. One of the private routes consists of the prescription panel page. The psychiatrist can choose an option to prescribe a patient from the patient's profile. Then, he will be redirected to the prescription panel, which only the psychiatrist can access.  Figure 15 shows the prescription panel interface. The names of both the patient and the psychiatrist will be dynamically added from their corresponding profiles. The psychiatrist will add the suspected category of the patient's state, and then, in the text area down below, he will write the detailed prescription. Later, when he presses the prescribe button, the whole form will be generated in a pdf format which will later be delivered to the patient's profile (Figure 16) with the psychiatrist's name and the issued date.

The article "Development of NLP-Integrated Intelligent Web System for E-Mental Health" was retracted in 2023. Reasons: signs of a paper mill; compromised peer review; unreliable results or conclusions.

Figure 16 shows the formatted pdf version of the prescription. From the prescription issue page, all the dynamic and inserted data by the psychiatrist will be extracted. Then, with all the extracted data, the pdf will be created in a previously fixed format.

### 4.4. User Dashboard

The user dashboard is the page where all the information and records related to the user's history will be displayed. It will be only visible to the user himself and the corresponding psychologist and authority. There, they will be able to see the previous meeting history, previously prescribed prescriptions, user's states, etc.  Figure 17 shows the meeting history of a user with the psychologists, and he can download that certain meeting's prescribed prescriptions easily.

### 4.5. Finding Psychiatrists

Registered users will be able to look for psychiatrists in the designated “Find Your Psychiatrist” panel. There, the patient will be able to view the profiles of various certified and registered psychiatrists. Then, he will choose between a number of them to connect with whom he will later talk and take all kinds of psychological services. After contacting a particular psychiatrist, the patient will access that psychiatrist's chatroom and have access to a scheduled video conference date. The “Find Your Psychiatrist” panel will constantly be updated with the latest enlisted and registered ones to keep up with the flow of patients willing to take service.  Figure 18 shows how a user can choose from a list of psychiatrists by his choice of details in that specific panel. There is a feasible search for psychiatrist features which will operate when the database has enough collections of psychiatrists.

### 4.6. Chatbot

The chatbot feature works as a module for now. It is a 3-layered Long Short-Term Memory deep neural network model built with TensorFlow and the Keras Application Programming Interfaces (APIs) for the Python interface. The Keras sequential API has been used for the three layers, dense, dropout, and activation, of the deep neural network. The dataset used for the chatbot is novel. After researching numerous well-established mental health condition analysis tests, MBTI test cases have been used to create a dataset for this paper. The MBTI, or Myers-Briggs Type Indicator, is one of the most prominent personality tests that has been used for this dataset. So, our dataset is one of a kind, and it can be improved further with other test cases in the future. This chatbot is well responsive and replies with relevant statements.

The article "Development of NLP-Integrated Intelligent Web System for E-Mental Health" was retracted in 2023. Reasons: signs of a paper mill; compromised peer review; unreliable results or conclusions.

Figure 19 displays the chatbot performing a MBTI test on the user. The JSON dataset for the chatbot is novel. There is no such open-source dataset available for testing. So, the dataset had to be made from scratch for this particular test [26]. MBTI test cases have 70 tests in total. The dataset implements the test cases to their full potential. Each test case has two possible answers. Based on the answers, the JSON dataset has 140 items for the MBTI test cases. An additional 5 items are for greetings and general conversation. So, the chatbot model is trained with 145 objects from the JSON dataset for 30 epochs. With more epochs, the model can be trained for more training and validation accuracy.  Table 1 shows chatbot accuracy and failure rates for the last three epochs.

This chat module serves as the primary assessment tool for the system. Through this conversational NLP chatbot, any user can self-assess his or her present personality condition. As the chatbot uses MBTI test cases, one of the most accepted test cases by professionals, the result of the chatbot will give a primary insight into the users' condition. Apart from self-assessment, this result will also be used in further steps of the system to deliver a better experience in the case of mental health support.

Figure 20 represents the graphical presentation of training data accuracy and validation data accuracy. After 30 epochs, the models get an accuracy of 91.42% for training and 86.04% for validation.  Figure 21 shows the graphical representation of training data loss of 0.2097 and validation data loss of 0.6378.

### 4.7. Video Conference Module

Figure 22 shows the video conference interface when two users are connected. Two devices on the internet can connect with each other through a video conference call. Users can call each other if they have each other's IDs; they can call each other just by copying their IDs. The further approach to this subsystem uses computer vision to recognize the participants' emotional state from their facial expressions. Then, this data is collected for further analysis.

The backend technology used here is WebSockets and socket programming. This server system runs on a Node.js runtime environment. React.js handles the client side. WebSockets simply provide an application with a means of smooth real-time communication via a simple API. In this system's case, the real-time video conference module is built with WebSockets and also with the help of socket programming. Socket programming here helps the system connect two devices to communicate with each other. Using computer vision, the system will use a deep learning model with which the video conference section will have a trained module. With it, the system will be able to detect one's emotion while he/she is in the video conference.

The article "Development of NLP-Integrated Intelligent Web System for E-Mental Health" was retracted in 2023. Reasons: signs of a paper mill; compromised peer review; unreliable results or conclusions.

By using this video conference module, users can be connected directly with the psychiatrist without having the hassle of going out for the meeting. It is also time-saving as they do not have to deal with the traffic jams by going outside to get the service. Also, it is more secure to keep the confidentiality of the meeting, and users can express their feelings more easily. It is also a cost-saver for both users and the psychiatrist.

### 4.8. Emotion Detector Module Using Computer Vision

In the emotion detection part, after we pass the user-side video through the model, it perfectly detects user emotions and changes the label according to the changing facial expression of the user.

The face detection label is blue and the emotion label is green, and it shows right upon the face of the user. The model can detect five types of different emotions. They are neutral, happy, sad, angry, and surprise.  Figure 23 shows that the emotion detection feature is working on users' facial expressions. It is detecting from the user's facial expression that the user's condition at the moment is happy.

### 4.9. Chat Forum Module

Figure 24 shows that a user is trying to enter a specific chat room based on his need. There are multiple channel choices in the room section. These rooms will serve the relevant purposes of different users at different times. The consequence is shown in Figure 25, where he enters and gets greeted by other participants there. He will be able to look at others' messages just like any other group chat. He will be able to see the participant users as well.

### 4.10. Payment Module

The website has a payment module, where if someone wants to receive any paid feature of the system, he will be able to make payments. The payment module is integrated with SSLCOMMERZ, which is the largest payment gateway aggregator in Bangladesh. For example, the mobile banking gateway has only been used on the websites of Bkash, Nagad, and Rocket. The system has used three APIs from SSLCOMMERZ to complete the integration, which are the create and get session, receive payment notification, and the order validation API.  Figure 26 shows the payment module section of the website where the user will be able to choose three different gateways to make the payments.

The article "Development of NLP-Integrated Intelligent Web System for E-Mental Health" was retracted in 2023. Reasons: signs of a paper mill; compromised peer review; unreliable results or conclusions.

### 4.11. Comparison Table with Other Existing Systems

Here, Table 2 shows the overall comparison of other existing models with the presented platform in this paper. If the system presented in this paper is compared with the existing platforms [4–6], it can be seen that the presented system has almost all the functionalities of already existing platforms, except the system in [2] which has online course offerings, which this system does not offer. However, the system presented has NLP conversational chatbot and emotion detection features on video conference, which is the most highlightable feature that makes it stand apart from the platforms presented in [4–6]. Also, in Figures 24 and 25, this system presents a chat forum feature, which is also a new feature that is missing in the already existing platforms.

## 5. Conclusion

During this pandemic, the world has observed the necessity of mental support and help among and surrounding themselves. Moreover, it is not always possible for the majority of the population to go out for the specific reason of meeting a psychologist. This web application is trying to implement the system's knowledge to give these people a platform to get the essential support for their condition. With a whole organized forum-based web application along with the help of NLP and computer vision, the system will be able to evaluate this problem efficiently. Features like facial expression recognition in video conferencing will be very beneficial in detecting a person's mental condition. Implementing cutting-edge real-time technologies has added a new dimension to evaluating the mental conditions of patients.

The research, as well as the system itself, has a lot of room to grow in the future. As the dataset for the NLP-based chatbot system is already made by one of the researchers, it always has a scope to get enriched with newer relevant data in the field of mental health. Technically, the web system is fairly current with cutting-edge technology; there is potential to convert the web system to a Progressive Web App (PWA) in the future for increased usability and reach. The web app can also feature a Short Message Service (SMS) system on a commercial level. Overall, this study offers a lot of promise for future expansion, both technically and in terms of research, and if commercialized, it has a lot of potential.

The whole system as a web app will be very convenient to both help seekers and professionals. People from anywhere will be able to get help and serve the purpose of mental health support through this web application. This will act as a one-stop solution to solve any mental health complications.

The article "Development of NLP-Integrated Intelligent Web System for E-Mental Health" was retracted in 2023. Reasons: signs of a paper mill; compromised peer review; unreliable results or conclusions.

## Figures and Tables

**Figure 1:** The system flow chart diagram.

**Figure 2:** The chatbot subsystem diagram.

**Figure 3:** The video call subsystem diagram.

**Figure 4:** The web forum subsystem diagram.

**Figure 5:** Use case diagram.

**Figure 6:** Socket.io-client initialization every time the page on the web app loads.

**Figure 7:** Call user function.

**Figure 8:** Answer call function.

**Figure 9:** Backend Socket.io structure for the chat module.

**Figure 10:** Backend service listening for chat messages.

**Figure 11:** Backend configuration for the video call system.

**Figure 12:** The home interface.

**Figure 13:** Psychologist authentication.

**Figure 14:** Regular user authentication.

**Figure 15:** Prescription form.

**Figure 16:** Demo prescription.

**Figure 17:** User's meeting history with prescription.

**Figure 18:** Finding psychiatrist.

**Figure 19:** Mental condition evaluation.

**Figure 20:** Graphical representation of training data accuracy and validation data accuracy.

**Figure 21:** Graphical representation of training data loss and validation data loss.

**Figure 22:** Video conference interface (users connected).

**Figure 23:** Showing the emotion detection of the user.

**Figure 24:** User joining a channel.

**Figure 25:** User chatting in a specific channel.

**Figure 26:** Payment section.

**Table 1:** Chatbot accuracy and failure for last three epochs.

Epoch	Loss	Accuracy
28/30	0.3765	0.9036
29/30	0.2924	0.9724
30/30	0.2097	0.9142

**Table 2:** Comparison table with other papers.

Features	Ref [4]	Ref [5]	Ref [6]	This system
Video conference	No	No	Yes	Yes
NLP chatbot	No	No	No	Yes
Community	No	No	No	Yes
Teletherapy	Yes	No	Yes	Yes
Condition evaluation	No	No	No	Yes
Online course	Yes	No	No	No
Find psychiatrist	No	Yes	No	Yes
Registration	Yes	Yes	Yes	Yes
Emotion detection	No	No	No	Yes
Chat forum	No	No	No	Yes

## Data Availability

The data utilized to support these research findings is accessible online at https://www.kaggle.com/abid0801/mbti-personality-test-cases.
